# A Context-Aware MRIPPER Algorithm for Heart Disease Prediction

**DOI:** 10.1155/2022/7853604

**Published:** 2022-07-11

**Authors:** Saad Almutairi, S. Manimurugan, Naveen Chilamkurti, Majed Mohammed Aborokbah, C. Narmatha, Subramaniam Ganesan, Riyadh A. Alzaheb, Hani Almoamari

**Affiliations:** ^1^Industrial Innovation and Robotics Center, Faculty of Computers and Information Technology, University of Tabuk, Tabuk, Saudi Arabia; ^2^Department of Computer Science and IT, La Trobe University, Melbourne, Australia; ^3^Department of Electrical and Computer Engineering, Oakland University, Rochester, NY, USA; ^4^Faculty of Applied Medical Sciences, University of Tabuk, Tabuk, Saudi Arabia; ^5^Faculty of Computer and Information Systems, Islamic University of Madinah, Medina, Saudi Arabia

## Abstract

These days, mobile computing devices are ubiquitous and are widely used in almost every facet of daily life. In addition, computing and the modern technologies are not really coexisting anymore. With a wide range of conditions and areas of concern, the medical domain was also concerned. New types of technologies, such as context-aware systems and applications, are constantly being infused into the medicine field. An IoT-enabled healthcare system based on context awareness is developed in this work. In order to collect and store the patient data, smart medical devices are employed. Context-aware data from the database includes the patient's medical records and personal information. The MRIPPER (Modified Repeated Incremental Pruning to Produce Error) technique is used to analyze and classify the data. A rule-based machine learning method is used in this algorithm. The rules for analyzing datasets in order to make predictions about heart disease are framed using this algorithm. MATLAB is used to simulate the proposed model's performance analysis. Other models like random forest, J48, CART, JRip, and OneR algorithms are also compared to validate the proposed model's performance. The proposed model obtains 98.89 percent accuracy, 96.76 percent precision, 99.05 percent sensitivity, 94.35 percent specificity, and 97.60 percent f-score. Predictions for subjects in the normal and abnormal classes were both accurate with 97.38 for normal and 97.93 for abnormal subjects.

## 1. Introduction

Context awareness originated as a term from ubiquitous computing, which is turning into a reality that highlights the integration between the data space and the physical space. With its assistance, individuals could receive and process data anywhere and anytime through a device that can link any Internet. Therefore, it can lessen the difficulty of utilizing the device and make individuals' lives simpler and progressively effective. The environment of user in ubiquitous computing, for example, the location or terminal equipment, is continually changing, which is called context. As part of the central zones of ubiquitous computing, context-aware computing has become increasingly very well known among people. Numerous authors have described context according to their comprehension with an exertion to review an extensive basic idea of the context [1]. Schilit and Theimer utilized the term context awareness in 1994 to refer to context as location, identities of objects and nearby people, and changes to those objects. The term context has been sorted into two classes (logical and physical) [2]. Physical context could be decided through hardware sensor and logical context was provided either through the user's feedback or by observing their communications with the services accessible, for instance, by monitoring or reviewing the user's profile, working schedules, activities, and composing movement. Most research around there utilizes physical sensor for movement, sound, touch, temperature, light, and of course location. The logical sensor though gives associated data by reading user's data from public website pages and different archives and furthermore reviews user's information (interaction) dependent on this interaction target publicizing [2].

A context can be various elements or factors such as location, user identity, time, activity, current task, environment, and hardware. Context awareness means that one can utilize context data. A system was context-aware if that it could extricate, decrypt, and use context data and modify their performance to the present context of usage. The name context-aware computing was generally perceived through those performing in context-aware, where it was considered that context was a source in its attempt to distribute and directly combine computer advancement into our lives. Context-aware systems can modify their activities dependent on the present context. This likewise expands adequacy by considering environmental context. CAS observes the condition constantly and proposes reasonable recommendations to users through which they could make important actions [3].

The context-aware healthcare system helps hospitals to enhance performance efficiency by incorporating real-time contextual data into the actual workflow like the locations and current conditions of medical devices and employees. It also allows access to environmental data in order to deliver the best possible patient experiences. The solution supports both real-time asset monitoring and event-driven tracking, with real-time tracking moving across the surrounding and event-driven tracking existing and entering regions. The primary goal of healthcare systems must be to safeguard and maintain the security of patient data. In addition, the use of context is critical in interactive frameworks where the user's data changes frequently, such as that in portable and ubiquitous computing (Figure 1).

Some of the previous works made use of several methodologies for applications in a variety of contexts and made use of numerous kinds of sensors, highlighting both their capabilities and their limitations. The difficulty in mapping the patient's context from many situations and sensors, all of which use distinct communication protocols, leads to a challenge in defining the patient's context awareness with a high degree of precision. As a result, a variety of approaches to the consolidation of data as well as modes of reasoning can be analyzed.

### 1.1. Context-Aware in Healthcare

The combination of Internet and the medical domain is a progressive innovation, with present research aiming at using computing to support in training among the medical sectors. The smart clinical devices market was predicted to reach above 126 billion dollars profit by the year 2028 while smart wearable devices intended to be extensively utilized to accomplish enhanced health, quality of life, and protection of people. Moreover, due to their capability of aiding real-time constant observance of patient's data, such devices also make context-aware mobility significance to enhance overall condition of medical care. Context-aware system (CAS) is a system that can adjust its activities to context changes without unequivocal user intercession. The CAS platform should unequivocally be presented by its component's functionalities, context data, and the control activity and furthermore provides services to users utilizing context data where pertinence relies upon the user's operation. In this way, a context-aware domain could be intended middleware support that permits the exchange of environmental data out of the minimum infrastructure range to a more significant range for definition and decision. This multilayered design was common for the cloud computing sequence that permits setting the middleware layer as a major aspect of a sensor-cloud interface in the layer of PaaS (Platform as a Service) [4].

Context-aware systems also play an important role in healthcare systems, whereby automatically distinguishing a patient from the rest of the surroundings, recording the various events associated with a specific patient, keeping track of the various services provided in a specific location, and providing the necessary documentation are some of the important functionalities that must be encountered by the system. There is also the extra obligation on the system to keep the patient's and healthcare professional's information secure and safe. Security is also required for any equipment used by healthcare institutions. As a result, healthcare systems cannot be viewed as a separate system from the rest of the technological systems; rather, they are a sociotechnical system that is dependent on the collaborated results of the communications among the technology and user. Context awareness aids in the more precise diagnoses of the observed patient's health problems. It can recognize behavioural patterns and so make more exact conclusions about people and their surroundings. Adaptation, personalization, and proactivity are the three most essential advantages of context awareness. The following was a breakdown of the three advantages.

Adaptation focused on tailoring the services or information to the user's present situation. A specific example is when the system in issue adjusts the data that it delivers based on networks and device contexts, like speed of connection and resolution of display. Personalization is the process of customizing the system to individual users, where each user sees the framework differently. Personalization was according to the individual user's choices, habit, abilities, duties, and so on. The data or, more accurately, the degree of detail at which information was supplied to doctors, i.e., in Healthcare Monitoring System, was plainly different from that received to patients or caretakers.

Proactivity was considered with providing services for the users based on forecasts of future circumstances. When it comes to Healthcare Monitoring Systems, proactivity is critical in producing really useful and promising solutions. There are several examples and user cases. For example, being proactive and determining health issue situations aid in the discovery of these concerns at the early stages, which frequently enhances the likelihood of averting or, at the very least, minimizing the harm caused by the health issues. Another situation or user case in which proactivity aids in the prediction of diseases-causing mutation induced by genetical alterations in the genomes was likely to get molecular effects. From the most recent decade, the CAS is targeted around web applications and desktop computing in the Internet of Things (IoT). Because of advanced sensor innovations, sensors are getting stronger, less expensive, and less in size. In this present world, there are numerous sensors and eventually these sensors create a lot of information, for example, big data. In case if we dissect, interpret, and comprehend the information which collected that information may not produce important data. Context-aware computing plays a significant part in handling this task, for example, mobile and pervasive, which would be effective in the IoT model also. This enables us to save the context data associated with sensor information, so the interpretation should be possible more effectively and genuinely and furthermore context makes it simpler to execute machine-to-machine interaction as it is the core component in the IoT condition [5].

Heart disease is one of the most critical and difficult health problems in the modern world. Heart disease reduces blood vessel function and causes coronary artery infections, both of which weaken the patient's body, especially in adults and the elderly. According to the WHO, heart diseases are the leading cause of death globally. In 2019, an estimated 17.9 million people died from heart diseases, accounting for 32% of total worldwide mortality. Stroke or heart attack caused 85 percent of these fatalities. More than three-quarters of all heart disease deaths occur in low- and middle-income countries. Heart diseases are responsible for 38% of the 17 million premature deaths (before the age of 70) caused by noncommunicable disease in 2019. Most heart disease can be prevented by addressing behavioural risk factors such as cigarette use, poor diet and obesity, inactivity, and excessive alcohol use. It is critical to detect heart disease as soon as possible so that therapy with counselling and medicines may begin. Heart diseases are a kind of heart and blood vessel disease. Among these, there are cerebrovascular disease, coronary heart diseases, peripheral artery diseases, congenital heart diseases, rheumatic heart diseases, deep vein thrombosis, and pulmonary embolism [https://bit.ly/35qpAGG].

Context awareness performs a significant role in the concept of Internet of Things, as it provides rich contextual knowledge that can make the system perform more effectively. Since every context of healthcare is different, it is important to determine an adequate context-aware architecture for IoT healthcare applications. In this work, a context-aware healthcare method based on the application of IoT was proposed. Smart medical devices were utilized to collect and retain patient data, which was stored in a database. The database contained context-aware data, such as the names, addresses, and medical histories of the patients. A rule-based machine learning technique, a modified RIPPER algorithm, was utilized to analyze and classify the data. The rules for analyzing data for the prediction of heart disease were developed using this algorithm. The remaining part of this research is presented in following sections: Section 2 discusses the related works, Section 3 presents the proposed methodology, Section 4 presents the performance analysis, and Section 5 presents the conclusion and future extension of the research.

## 2. Related Works

Yousef presented an analysis of healthcare monitoring framework and its offerings on the IoT platforms. Many functions that exist in healthcare systems have been described and modelled. In addition, this work aimed to establish and propose the general frameworks for the development and design of contexts-aware healthcare monitoring framework in IoT domain. The essential elements of healthcare monitoring framework, as well as their relationships, were discovered and modelled in such a model. The work also emphasized the importance of the AI sectors in tackling robust context-aware healthcare monitoring. This framework was built on a distributed layer architecture, with distinct components implemented across the physical layers, cloud platform, and fog platform [1].

Mohamed et al. presented a novel decision-making paradigm focused on an IoT method for identifying and tracking type 2 diabetes patients. Wireless BAN was used to track changes in the user's body symptoms, and a smartphone phone interface was used to record social interactions. Since it was necessary to enhance the decision support schedules for the accurate predictions of type 2 diabetes issues, the hybrid approach focusing on type 2 neutrosophic with the VIKOR process was proposed in this analysis. The performance of this model was satisfactory and the accuracy could be improved by using advanced approach [6]. Abdur et al. proposed a knowledge discovery-based approach that enabled a context-aware system to change its behaviour in real time by analyzing large volumes of data produced in ambient assisted living frameworks and stored in the cloud databases. The proposed model allowed big data research within a cloud setting. It first analyzed the dynamics and patterns in a particular patient's records, along with the associated odds, and then used the information to learn proper irregular conditions. The results of this learning approach were then used in context-aware decision-making scheme for the patient. This model can be improved with more context domains [7]. Deeba and Saravanaguru proposed a model for monitoring signs and health conditions of elderly people. The data from the system was observed by the caregivers for identifying the daily activities through IoT. A fuzzy logic controller was designed from the initial stage of data collection, data processing, filtering, and accumulating it into contextual data and reasoning for identifying the elder people's health conditions [8]. Nourmohammadi-Khiarak et al. proposed a novel hybrid technique for heart diseases diagnosis using optimization method in feature selections. This analysis mainly focused on the features selection enhancement and reducing the features count. In this analysis, imperialist competitive algorithm with metaheuristic technique was proposed to choose essential features of the heart diseases and the K-nearest neighbour technique was utilized for the classification. This model could enhance the features selection technique for missed and incomplete data [9].

Daniel designed a context-aware system to assist healthcare providers in home-based caring environments. A reliable NFC authentication scheme was used, which creates a secure channel by encoding sensitive contextual data during data transmissions. Using a context-aware gateway node, this system performs authentications and authorization for accessing a specific patient's data. The proposed solution aimed to improve healthcare data access and safe data delivery while protecting users' privacy. This research provided a foundation for physicians to develop different smart treatment alternatives and for home-based care [10]. Deeba and Saravanaguru proposed a Smart Home Caregivers System (SHCS) capable of collecting real-time patient's heart rate and oxygen leakage in abnormal and normal patient's condition observed through MQ6 sensor. The data sensed was transmitted to the base station, where it was controlled by caregivers via PC or mobile device. This method was carried out by either wired or remote users using REST web services [11].

Based on fuzzy logic, Byung et al. presented context-aware healthcare model for disease reasoning. It was made up of two modules: fuzzy-based disease reasoning model (FDRM) and the fuzzy-based context-aware model (FCAM). The FCAM calculated the correlations coefficients and supports among the conditional attributes and the decision attributes and produced fuzzy rule based solely on the conditional attributes with the highest correlation coefficients and supports. Based on the results performed with a SIPINA mining method, the average accuracy of fuzzy rules dependent on correlations coefficients and supports (FRCS) and enhanced C4.5 was 0.84 and 0.81, respectively. That is, as correlated to the enhanced C4.5, the FRCS reduced the rules produced while improving accuracy of rules [12].

Haya Elayan et al. presented a digital twin framework for smart context-aware healthcare systems in order to improve the quality of care provided to patients and the procedures involved in providing healthcare. This digital twin model used Internet of Things (IoT) devices, data analytics, and artificial intelligence over the course of three stages and generated a patient's virtual replica, making it easier for medical professionals to work together and supporting patients with similar conditions. As a result, a classifier model for ECG heart rhythms was developed with the use of machine learning in order to diagnose heart disease and identify cardiac abnormalities [13].

Sujaya and Rashmi proposed a context-aware automated activity monitoring system with the purpose of continuously monitoring the physiological state of old persons as well as changes in their behavioural activity. In this system, sensory information was gathered using a wide array of sensors in various locations. The health of elderly people was predicted by employing signal processing, machine learning approaches such as support vector machines (SVM), and cloud-assisted context-aware on-demand and proactive healthcare support. All of this was done based on collected sensory data [14, 15].

By analyzing these related works, it was found that most of the researches used the sensors as the IoT device for collecting biosignal data in terms of digital format. Those data are stored in cloud for easy accessing and data storage. Mostly, machine learning techniques are used for the classification of medical data. A lot of limitations have been analyzed in these related works such as improper dataset selection, which failed to acquire some important data related to heart disease using sensors, poor classification performance, and misclassified results. By keeping this in mind, a proper context-aware based heart disease prediction model is proposed in this research. Finally, all these works failed to focus on the data security and privacy, which could support the patients' trust and support on these future technologies.

## 3. The Proposed Methodology

In this work, a context-aware healthcare method based on the application of IoT was proposed. Smart medical devices were utilized to collect and retain patient data, which was stored in a database. The database contained context-aware data, such as the names, addresses, and medical histories of the patients. A rule-based machine learning technique, a modified RIPPER algorithm, was utilized to analyze and classify the data. The rules for analyzing data for the prediction of heart disease were developed using this algorithm. Based on the classification results, the prediction of the heart disease was performed (Figure 2). The smart medical wearable devices based on body sensor network are used for the computation of patient's physiological medical data (i.e., heart rate and temperature). The data from these devices are stored in the cloud platform for data storage. The stored data can be further managed or used by the user or the medical centres for analyzing the patient's health conditions. By using specific application, the patient can be monitored from remote places via Internet through smartphones or PCs. The block diagram of the model was shown in Figure 2. The proposed algorithm is discussed as follows.

The IoMT devices and wearable devices are considered as the IoT devices. They are equipped to accumulate the patient's data from remote areas. These data are collected as patient's information that are accumulated using IoT devices connected or equipped with the human body.

### 3.1. RIPPER Algorithm

The rule-based machine learning can be detailed as the basic concept description. The RIPPER algorithm is one of the most widely used techniques. Comparing to various algorithms, this technique has more benefits; it could be comprehended with ease, with generated rules in the form of If-Then format, implying that the model is entirely interpretable. The RIPPER algorithm is a rule-based classification algorithm that produces a rule-based classifier model, which is a collection of IF-THEN rules derived straight from the training dataset; thus the name is “direct process.” It can be utilized for multiclass and binary classifications. The RIPPER algorithm's core framework was split into two types: optimization rules and generation rules. The generation type is the two-layer loops in which the outer loop produces the rule and applies it to the rule base next to pruning, while the inner loop includes one antecedent to the rule at once. Based on the Base's Rules (BR), the optimization type creates alternate rules, and the minimum description length (MDL) criteria were utilized to pick the right rule and attach it with rule base [16]. This algorithm goes through four stages.

*Growth.* During this process, a rule was created by greedily applying features to the rule before it passes the stopping criterion.

*Pruning.* Throughout this process, every rule was pruned and rendered shorter by eliminating repetition and reducing the duration of previous rules, allowing the rule to improve.

*Optimization.* The initial prune and growth process creates rules from an empty rule set. The optimization phase makes use of the rules created during the initial pruning and growth stages and attempts to create new rules from the rule set. The rules can be additionally optimized with the following.

- Add features to the initial rule using the greedy approach (i.e., depth initial search).
- Follow the growth and pruning process; a new rule set is created.

*Selection.* At the selection process, the best rules were held and the rest of the rules are removed from the system. The specifications of this algorithm are as follows: *D* dataset is used as input ((1) and (2)).

Step 1: split the dataset *D* into individual growth sets *Gro* and prune set *Pru*.
Step 2: the growth set *Gro* was utilized at this point as dataset. The growth rule starts with no rules, and every time an appropriate combination of potential features and thresholds is chosen as the antecedents would be included to the rules. The information gain was utilized as the evaluation criterion:
  (1) $$\begin{array}{c} IGN=\text{cover}\left(\log_{2}\;rt\prime -\;\log_{2}\;rt\right). \end{array}$$
Cover is the number of positive instances that were covered since adding the antecedents to the rule, *rt*′ was the proportion of positive instances in the data covered using the rule, and *rt* is not considered. The iteration of including antecedents would continue until the *Gro* was empty.
Step 3: the pruning process utilizes the pruning set *Pru* to measure the rule's generalization capacity. Begin with the past thing added and eliminate an antecedent in the rule. When pruning, the metric was
  (2) $$\begin{array}{c} T=\frac{p-n}{p+n}. \end{array}$$
*p* was positive instances covered by the rule in *Pru*, *n* was negative instances covered by the rule in *Pru*, and the point of the calculation was to increase the precision of the pruned set.
Step 4: after pruning the rule, it was tried to be included to a rule base. The inclusion would fail if the number of instances covered by the rule was too limited or the precision was too poor. If the rule was effectively included, the instances covered will be removed from the *D* [17].

### 3.2. MRIPPER Algorithm

The RIPPER algorithm for rule induction was implemented as a replacement for the Incremental Reduced Error Pruning (IREP) algorithm. About the fact that the fundamental ideals remain similar, modified RIPPER strengthens IREP in certain details and was also capable of dealing with multiclass issues. A single MRIPPER rule was made up of a consequent and an antecedent part. The antecedent part was a predicate (selector) conjunction, and the consequent part was a class assignment. MRIPPER learns those rules greedily, using a divide-and-conquer approach. The training data are classified by class terms in increasing order based on the respective class frequencies prior to the learning process. The rules for the initial m-1 classes are then learned, beginning with the smallest. When the rule was established, the instances concealed by that rule are excluded from the training data, and this process was replicated till no instances from the target classes remain. After that, the algorithm moves on to the next class. Finally, as MRIPPER discovers that there are no more rules to learn, a default rule (with an empty antecedent) was applied for the last class. Single-class rules are learned before either all positive instances were concealed or the last rule applied was “too difficult.” The last feature was applied in terms of overall description length: the stopping criteria were met if R's description length was quite longer than the shortest description length found so far as represented in the algorithm [18].

### 3.3. The Proposed Algorithm

 
*procedures BUILDSET (P, N)*
 
*P=* *positive samples*
 
*N* *=* *negative samples*
 
*Rule Set* *=* *{}*
 
*DL* *=* *Description length (Rule Set, P, N)*
 
*while P {}*
 
*//Grow and prune a new rule*
 
*split (P, N) into (Gro P, Gro N) and (Pru P, Pru N)*
 
*Rule* *=* *Gro Rule (Gro P, Gro N)*
 
*Rule* *=* *Pru Rule (Rule, Pru P, Pru N)*
 
*add Rule to Rule Set*
 
*if Description Length (Rule Set, P, N)* *>* *DL* *+* *11 then*
 
*//Prune the whole rule set and exit*
 
*for every rule R in Rule Set (considered in reverse order)*
 
*if Description Length (Rule Set {R}, P, N)* *<* *DL then*
 
*delete R from Rule Set*
 
*DL* *=* *Description Length (Rule Set, P, N)*
 
*end if*
 
*end for*
 
*return (Rule Set)*
 
*end if*
 
*DL* *=* *Description Length (Rule Set, P, N)*
 
*delete from P and N all instances covered by Rule*
 
*end while*
 
*end BUILDRULESET*
 
*procedure OPTIMIZERULESET (Rule Set, P, N)*
 
*for every rule R in Rule Set*
 
*delete R from Rule Set*
 
*U Positive* *=* *instances in P not covered by Rule Set*
 
*U Negative* *=* *instances in N not covered by Rule Set*
 
*split (U P, U N) into (Gro P, Gro N) and (Pru P, Pru N)*
 
*Rep Rule* *=* *Gro Rule (Gro P, Gro N)*
 
*Rep Rule* *=* *Pru Rule (Rep Rule, Pru P, Pru N)*
 
*Rev Rule* *=* *Gro Rule (Gro P, Gro N, R)*
 
*Rev Rule* *=* *Pru Rule (Rev Rule, Pru P, Pru N)*
 
*select best of Rev Rule and Rep Rule and add to Rule Set*
 
*end for*
 
*end OPTIMIZERULESET*
 
*procedure RIPPER (P, N, k)*
 
*Rule Set* *=* *BUILDRULESET (P, N)*
 
*repeat k times*
 
*Rule Set* *=* *OPTIMIZERULESET (Rule Set, P, N)*
 
*return (Rule Set)*
 
*end RIPPER*

### 3.4. Rule Set

  Rule 1: if (Thallium was less) and (Chest pain was typical angina) hence (No heart disease)
  Rule 2: if (Thallium was less) and (Chest pain was atypical angina) hence (No heart disease)
  Rule 3: if (Thallium was less) and (Chest pain was nonangina) hence (No Heart disease)
  Rule 4: if (Thallium was less) and (Chest pain was asymptomatic) and (Vessel was less) hence (No Heart disease)
  Rule 5: if (Thallium was less) and (Chest pain was asymptomatic) and (Vessel was higher) hence (Presence of Heart disease_2)
  Rule 6: if (Thallium was higher) and (vessel was less) and (No angina) hence (No Heart disease)
  Rule 7: if (Thallium was higher) and (vessel was less) and (has angina) hence (Presence of Heart disease)
  Rule 8: if (Thallium was higher) and (vessel was less) hence (Presence of Heart disease_2)
  Rule 9: if (family history was true) hence (Presence of Heart disease_1)
  Rule 10: if (medical record was true) hence (Presence of Heart disease_1)
  Rule 11: if (family history was true) and (medical record was true) hence (Presence of Heart disease_1)

The rule set for the algorithm discussed is framed based on the medical condition of the patient regarding the prediction of heart disease prediction. The rule set is framed from the conditions related to the causes of heart disease as shown in Table 1. Each attribute represented in the table has the range based on the condition of description. According to the ranges, the disease condition will be predicted with the rule set framed for context-aware system. The context database collects the context-aware data from the input which is medical records, personal information, and physiological data of the patient. Based on the context analyzer and context reasoning, the rule set is framed and analyzed. The data from the context database is processed by the proposed algorithm for the classification. For experimental analysis, the Cleveland dataset is implemented in this research for evaluation.

## 4. Performance Analysis

The proposed model's performance analysis was experimented in the MATLAB and Simulink tool. The experiment was carried out on a 64 bit CPU, i5 processor operating on Windows 10, with 8 GB RAM, using the MATLAB and Simulink tool R2017a. The data classification is significant in this analysis. The proposed classifier classifies the data for the prediction of heart disease, whose result will be in the form of absence or presence of disease. The results are carried out using the dataset and various classification parameters like accuracy, recall, precision, and F-measure. For classification, the benchmark dataset is classified using rule-based machine learning classifier called modified RIPPER algorithm. In this analysis, the heart disease prediction is the main work concentrated and the prediction model can be used to perform prediction for any serious disease by using the different dataset in the process.

### 4.1. Dataset Description

For the heart disease prediction and classification, Cleveland dataset from UCI repository was utilized in this research, available in public database. Each dataset has its very own instances and attributes; that Cleveland dataset is used for training which has 76 attributes and 303 records. But, only 13 attributes in dataset were utilized for this analysis and experiment as represented in Table 2 [20].

The data sample from the Cleveland dataset is shown in Table 3. It represents the data of two patients collected in the form of numerical value. Here, the medical term data are represented numerically according to the description presented in Table 2. Performance metrics such as accuracy, sensitivity, specificity, precision, and F-measure are used to evaluate the proposed model's performance. These metrics are calculated using true positive (Tpos), true negative (Tneg), false positive (Fpos), and false negative (Fneg) measurements.

In general, the accuracy of data is determined by how it was obtained. It was calculated by comparing various metrics from the same or different source

(3) $$\begin{array}{c} \text{Accuracy}=\frac{\text{Tpos}+\text{Tneg}}{\text{Tpos}+\text{Fpos}+\text{Tneg}+\text{Fneg}}\%. \end{array}$$

Precision, also known as positive predictive values, was the probability that a person with a positive screening test truly had the disease. The precision may be determined, as stated by

(4) $$\begin{array}{c} \text{Precision}=\frac{\text{Tpos}}{\text{Tpos}+\text{Fpos}}. \end{array}$$

Recall or sensitivity measures the ability of detecting a patient at risk for heart disease and is stated as

(5) $$\begin{array}{c} \text{Recall}=\frac{\text{Tpos}}{\text{Tpos}+\text{Fneg}}. \end{array}$$

Specificity is measured by dividing the total number of negatives by the number of genuine negatives, as shown in the following equation. The highest specificity is represented by 1.0, while the lowest is marked by 0.0:

(6) $$\begin{array}{c} \text{Specificity}=\frac{\text{Tneg}}{\text{Tneg}+\text{Fpos}}. \end{array}$$

The F-measure, which is defined as the weighted harmonic mean of test precision and recall, assesses test accuracy. The accuracy does not take into account how the data is disseminated. As a result, the F-measure is utilized to accurately manage the distribution problem

(7) $$\begin{array}{c} \text{F}-\text{Score}=\frac{2\text{Tpos}}{2\text{Tpos}+\text{Fpos}+\text{Tneg}}. \end{array}$$

Tpos, true positive, is proper prediction on healthy classes.

Tneg, true negative, is proper prediction on abnormal classes.

Fpos, false positive, is improper prediction on healthy classes.

Fneg, false negative, is improper prediction on abnormal classes.

From the dataset, the selected data are analyzed and classified by the proposed MRIPPER algorithm. Five healthy samples and five abnormal (heart disease) samples are used for the experiment in this research. The subjects 1–5 are classified as healthy class and 6–10 are classified as abnormal class from the dataset. The performance analyses of these ten subjects are computed and tabulated in Figure 3 and 4 representing the graphical representation of performance analysis made on normal and abnormal subjects as shown in Table 4. Accuracy, precision, recall, specificity, and f-score are the parameters used in this research for the evaluation of performance.

Table 5 represents the comparison of the proposed algorithm's performance analysis with other existing algorithms. The proposed MRIPPER algorithm is compared with random forest, J48, CART, JRip, and OneR algorithms. The proposed approach obtained 98.89 percent accuracy, which was 1.2% to 4.8% higher than the other algorithms. Precision of the MRIPPER algorithm is 96.76%, which is 1.7% to 3.5% higher, recall or sensitivity is 99.05%, which is 1.2% to 4.8% higher, specificity is 94.35%, which is 0.8% to 4% higher, and f-score is 97.60%, which is 1.4% to 6.4% higher than the other algorithms. Overall, the proposed approach has attained 97.93 percent in predicting abnormal class and 97.38 percent accuracy for normal class subjects (Figures 5 and 6).

## 5. Conclusion

The use of context awareness in medical field is embedded with other domains like IoT and cloud computing. With the combination of integrating with these technologies, the developed application on context awareness system has many advantages over other methods. Different applications like health monitoring, analyzing diseases, and assisting on medications can be done on remotely with the combinations of these technologies. In this work, a context-aware healthcare method based on the application of IoT was proposed. Smart medical devices were utilized to collect and retain patient data, which was stored in a database. The database contained context-aware data, such as the names, addresses, and medical histories of the patients. A rule-based machine learning technique, a modified RIPPER algorithm, was utilized to analyze and classify the data. The rules for analyzing data for the prediction of heart disease were developed using this algorithm. Models like random forest, J48, CART, JRip, and OneR algorithms are compared for the validation of the proposed model. The proposed model obtains 98.89 percent accuracy, 96.76 percent precision, 99.05 percent sensitivity, 94.35 percent specificity, and 97.60 percent f-score. Predictions for subjects in the normal and abnormal classes were both accurate with 97.38 for normal and 97.93 for abnormal. In the future, to increase the performance of the proposed model, a feature selection algorithm can be implemented to select the best optimal features to classify based on the disease condition. Also, this research will focus on adding data security and privacy for the data to be shared and stored in the cloud database.

## Figures and Tables

**Figure 1:** General process of context-aware system.

**Figure 2:** Block diagram of the proposed model.

**Figure 3:** Performance analysis on normal subjects.

**Figure 4:** Performance analysis on abnormal subjects.

**Figure 5:** MRIPPER performance.

**Figure 6:** Comparison of performance with existing algorithms.

**Table 1:** Description of data used in rule set.

Type	Range	Description

Chest pain	1 to 4	Typical angina
		Atypical angina
		Nonangina
		Asymptomatic

Cholesterol	<197	Lower
	188–250	Medium
	217–307	Higher
	>281	Very higher

BP	<134	Lower
	124–153	Medium
	142–172	Higher
	>154	Very higher

Blood sugar	<120	No
	≥120	Yes

ECG	<0.4	Normal
	0.4–1.8	Abnormal
	>1.8	Hypertrophy

Thallium	3	Normal
	6	Fixed defect
	7	Reversible defect

Age	<35	Younger
	35–45	Middle
	40–58	Older
	>58	Very older

Gender	1	Male
	0	Female

Smoking (in years)	≤10	Lower
	>10	Higher

Drinking	0	No
	1	Yes

Family history (diabetes, hypertension, ...)	<1	No
	≥1	Yes

Medical records (diabetes, hypertension, ...)	<1	No
	≥1	Yes

**Table 2:** Descriptions of Cleveland dataset [19].

Medical term	Description

Age	Age (years)
Gender	1 = male; 0 = female
Chest pain	Types of chest pains: 1-typical angina, 2-atypical angina, 3-nonanginal pain, and 4-asymptomatic
Bps	Resting blood pressure (mm HG)
Chol	Serum cholesterol (mg/dl)
Fastbs	Fasting blood sugar>120 mg/dl: 0-False and 1-true
Continuous max heart rate measured	Exercises induced angina: 0-no and 1-yes
Thalac	Max heart rate obtained
ST	Depressions induced by exercises related to rest
Slopes	The slopes of the peak exercise segments: 1-upsloping, 2-flat, and 3-downsloping
Cal	Total major vessels coloured by fluoroscopy which ranged from 0 to 3
Thall	3-normal, 6-fixed defects, and 7-reversible defects
Classes	Diagnosis classes: 0-healthy and 1-presence of heart disease

**Table 3:** Sample of dataset.

Age	Sex	Cp	Trestbps	Chol	Fbs	Induced angina	Thalach	ST	Slope	Ca	Thall	Class

55	0	3	115	322	0	0	160	1.6	2	0	7	0
74	1	2	124	261	0	0	141	0.3	1	0	7	1

**Table 4:** Comparison of performance evaluation on normal and abnormal subjects using MRIPPER algorithm.

Class	Accuracy	Precision	Recall	Specificity	F-score

Healthy class	96.48	94.81	97.21	89.64	95.50
	97.26	95.20	98.43	90.26	96.85
	96.40	94.73	97.10	89.12	95.08
	97.91	95.08	98.43	91.35	96.32
	98.85	96.93	99.20	92.48	97.05

Abnormal class	98.97	94.99	99.62	91.95	97.37
	98.51	96.64	99.45	90.16	97.01
	97.32	95.82	98.35	89.78	96.95
	98.04	96.34	98.92	91.65	97.46
	96.85	94.75	97.45	89.51	95.68

**Table 5:** Comparison of performance analysis.

Algorithm	Accuracy	Precision	Recall	Specificity	F-score

J48	94.08	93.45	95.82	90.24	91.18
Random forest	95.56	93.83	94.20	91.70	93.55
CART	95.80	94.06	96.48	90.96	96.13
OneR	96.48	93.21	96.54	92.11	95.24
JRip	97.66	95.01	97.80	93.54	96.15
MRIPPER	98.89	96.76	99.05	94.35	97.60

## Data Availability

The authors confirm that the data supporting the findings of this research are available within the article.
